# Immune Subtype Profiling and Establishment of Prognostic Immune-Related lncRNA Pairs in Human Ovarian Cancer

This article has been retracted.

**DOI:** 10.1155/2022/8338137

**Published:** 2022-05-05

**Authors:** Xingling Wang, Jing Wang, Mingxin Yu

**Affiliations:** Department of Gynecology, Cancer Hospital of China Medical University, Liaoning Cancer Hospital & Institute, No. 44 Xiaoheyan Road, Dadong District, Shenyang, 110042 Liaoning Province, China

## Abstract

This study collected immune-related genes (IRGs) and used gene expression data from TCGA database to construct a molecular subtype of ovarian cancer (OV) based on immune-related lncRNA gene pairs (IRLnc_GPs). The relationships between molecular subtypes and prognosis and clinical characteristics were further explored. IRGs were acquired from the ImmPort database, and round-robin pairing of immune-related lncRNAs was performed. The NMF algorithm was used to identify molecular subtypes, and the immune score of a single sample was calculated through ESTIMATE, TIMER, ssGSEA, MCPcounter, and CIBERSORT. The relationship between molecular subtypes and immune microenvironments was identified. A hypergeometric test was used to test the lncRNA pairs among the OV molecular subtypes (C1 and C2 subtypes). The BH method was used to screen the different lncRNA pairs, and a predictive risk model was constructed and verified. Finally, correlation analysis between the risk model, immune checkpoint genes, and chemotherapy drugs was carried out. Based on IRLnc_GP to classify 373 OV samples of TCGA, the samples were divided into two subtypes, and the prognosis between the subtypes showed significant differences. The C1 subtype with a poor prognosis was more related to the pathways of tumor occurrence and development. We identified 180 differential lncRNA pairs between subtypes and constructed a prognostic risk model based on 8 IRLnc_GPs. In the independent dataset, the distribution of subtypes in functional modules was different and highly repeatable. There were significant differences in the molecular and clinical characteristics of the subtypes and the drug sensitivity of immunotherapy/chemotherapy. In conclusion, the risk model established based on IRLnc_GP can better evaluate the prognosis of OV samples and can also assess the effects of different drug treatments in the high- and low-risk groups, providing new insights and ideas for the treatment of OV.

## 1. Introduction

The annual incidence of OV ranks third among female reproductive system tumors in China, after cervical cancer and uterine corpus malignant tumors [1]. The incidence is increasing year by year, and new cases and deaths remain high. The mortality rate ranks first among malignant tumors of the female genital tract, reflecting that OV is highly malignant and seriously endangers women's health [2]. Globally, the incidence of OV in developed countries is 9.2 per 100,000, and that in developing countries is 5.0 per 100,000 [3]. In 2017, approximately 22,440 women in the United States suffered from OV, and 14,080 patients died of OV [4]. The ovarian anatomy is hidden, and early OV lacks significant clinical manifestations and no specific indicators [5]. Therefore, early detection and early diagnosis of OV are difficult. Thus, when discovered, the cancer is often in the late stage of the disease, with some patients even experiencing metastasis to the peritoneum or distant locations. Patients with advanced OV have high resistance to postoperative chemotherapy and poor treatment effects [6]. Therefore, research on the pathogenesis of OV, especially the molecular mechanism, is particularly urgent.

There are apparent differences in the expression profiles of lncRNAs in normal tissues and tumor tissues, and related studies have shown that lncRNAs can affect the biological processes of cell proliferation, apoptosis, and invasion through transcription and posttranscriptional regulation [7] and are tightly linked to the metastasis and development of tumors. Both cancer-promoting lncRNAs and cancer-suppressing lncRNAs are expressed in the body [8]. Under normal circumstances, the two participate in cell proliferation and differentiation and can reach a relative balance; however, under the action of cancer-promoting factors, the expression of lncRNAs will be abnormal and can lead to cancer [9]. With continuous in-depth research on the correlation between lncRNAs and tumors, the relationship between the two has gradually become apparent, which can provide directions for the diagnosis and treatment of various malignant tumors [10–12].

Cancer is a very complex disease, and its regulatory networks are even more complicated and changeable. Cancer cells have different characteristics from normal cells, including immortal proliferation, avoidance of apoptosis, and growth inhibition [13]. These characteristics are formed under the influence of factors such as heredity, epigenetics, and the cancer microenvironment [14]. In the molecular network regulation mechanism during the formation of cancer cells (especially the signal transduction networks of cell carcinogenesis), gene pairs, as important nodes and centers, participate in the transmission of oncogenic signals and promote the growth of cancer cells [15]. The study of global lncRNA gene pairs in cancer cells or tissues helps understand the relationship between genotype and phenotype to better discover the mechanisms of cancer occurrence and development between normal and abnormal cells or tissues. This study screened IRLnc_GP, which may act as a predictive role in cancer, and established molecular subtypes, which provide specific guidance and a research basis for cancer treatment.

## 2. Materials and Methods

### 2.1. Sources of Expression Profile Data and IRGs

Expression data and clinical follow-up information (OV patients) were acquired from TCGA database (December 17, 2020). The RNA-Seq data of TCGA-OV were processed in the following steps: (1) samples without clinical follow-up information or survival time or status information were removed; (2) Ensembl codes were converted to gene symbols; (3) the expression levels of multiple gene symbols and the midvalue data were determined. The preprocessed TCGA-OV had a total of 373 samples (Supplementary Table1); a series of samples were downloaded from the ImmPort database (http://www.immport.org) [16] which provided the recognized IRGS. The prognostic workflow related to the characteristics of immune gene-related lncRNA pairs in OV is shown in Figure 1.

### 2.2. Identification and Pairing of Immune lncRNAs

We downloaded the latest version of the GTF file from the GENCODE website (https://www.gencodegenes.org/) [17], divided the expression profiles from TCGA into mRNA and lncRNA according to the annotations, and calculated the coexpression of each immune gene and lncRNA Pearson's correlation coefficient (value > 0.7) and *p* value (*p* < 0.05). Ultimately, 905 IRLnc_GP met the requirements, including 260 lncRNAs and 246 IRGs (Supplementary Table2).

The immune-related lncRNA cycles were matched. It was assumed that C was equal to lncRNA A plus lncRNA B to construct a 0 or 1 matrix; if the expression level of lncRNA A was higher than lncRNA B, C was defined as 1; otherwise, C was defined as 0. Then, the constructed 0 or 1 matrix was further screened, and the lncRNA pairs whose proportions of 1 lncRNA pair were 1 in all samples were higher than 50%.

### 2.3. Nonnegative Matrix Factorization(NMF) Algorithm and LASSO Analysis

The NMF method was used to select the standard “brunet,” and 100 iterations were performed. Cluster *k* set, 2~10, R package “NMF” [18], was used to determine the common member matrix (each subcategory^Minimum^ = 10). The optimal number of clusters was determined in terms of indicators such as cophenetic, dispersion, and silhouette (cluster = 2). The cophenetic correlation coefficient was acquired based on the consensus matrix.

It was based on a more refined model by building a penalty function to compress and set some coefficients to zero simultaneously, which was defined LASSO (most minor absolute shrinkage and selection operator) method. Then, the advantage of subset shrinkage was preserved. LASSO is a biased estimate for handling data with multicollinearity. The R package “glmnet” [19] was used to perform LASSO Cox regression analysis.

### 2.4. Functional Enrichment Analyses

In order to observe the functional differences between different subtypes, we downloaded hallmark gene set [20] from the msigdb database, used the GSEA software [21] for functional enrichment analysis, and set *p* < 0.05 and FDR < 0.25 as thresholds to screen significantly enriched pathways. The analysis of the enrichment pathways of Gene Ontology (GO) and Kyoto Encyclopedia of Genes and Genomes (KEGG) were conducted utilizing the R program WebGestalt R [22] for genes so as to detect the GO terms that displayed overrepresentation in 3 distinct categories (cellular component, molecular function, and biological processes) and KEGG pathway. With respect to all analyses, a FDR of less than 0.05 was regarded to indicate significance.

#### 2.4.1. Immune Infiltration Analysis

In order to evaluate the difference of immune microenvironment of different molecular subtypes, we first calculated the immune and matrix scores of each patient by using the R software package estimate [23] to evaluate the difference of immune infiltration between different subtypes and used the timer online platform (http://cistrome.org/TIMER/) [24] to evaluate the composition proportion of six immune cells in each patient. We also used ssGSEA method [25] to evaluate the score of immune cell infiltration in 28 and used R software package MCPcounter [26] to calculate the score of immune cell infiltration in 10 in each patient, CIBERSORT [27] was also used to evaluate 22 immune cell infiltration components of each patient, and the differences of immune cell infiltration in different subtypes were systematically compared based on the above four methods.

### 2.5. Statistical Analysis

The R (v.3.6.0) software was performed for statistical analysis. The Kaplan-Meier method was used to draw the survival curve and compared it with the log-rank test. The *p* values of the two sides were calculated. *p* < 0.05 is statistically significant.

## 3. Results

### 3.1. Identification of Molecular Subtypes

First, TCGA lncRNA pair data were analyzed by single-factor Cox regression using the coxph function in R and 426 lncRNA pairs (Supplementary Table3) related to the prognosis of OV (*p* < 0.01) were obtained. Then, nonnegative matrix factorization (NMF) was used to aggregate the OV samples. In theory, when each sample is clustered into one class, the value is the smallest, but such results were not available, so they needed to be used in conjunction with other indicators (Figures 2(a) and 2(b)). We further analyzed the prognostic relationships between the two groups, and the results indicated significant differences in OS and PFS times between the C1 and C2 groups (Figures 2(c) and 2(d), log-rank *p* < 0.01); the prognosis of the C1 subtype was poor.

### 3.2. Tumor Microenvironment (TME) Assessment and GSEA Pathways Enriched in Molecular Subtypes

To identify the relationships between the immune microenvironments of the two molecular subtypes, we used ESTIMATE, TIMER, ssGSEA, MCPcounter, and CIBERSORT to calculate the immune scores of each sample. We then compared them (Figures 3(a)–3(e)). The outcomes indicate that Tregs were significantly higher in C2 than the C1 subtype (*p* < 0.001). The stromal score and ESTIMATE score were higher in C1 than the C2 subtype (*p* < 0.001).

GSEA in the OV dataset was adopted to analyze the remarkably enriched pathways in the C1 and C2 subgroups. The selected gene set was HALLMARK, which contains 50 validated HALLMARK pathways. The GSEA input file contained the expression profile data from TCGA, the sample label of molecular subtype labeling, and the sample label for labeling the sample as a C1 group or a C2 group. The threshold for the selection of enriched pathways was *p* < 0.05 and FDR < 0.25, from which we obtained the significantly enriched pathways (Supplementary Table4) and found that there were more enriched tumor-related pathways in the C1 subtype group, such as epithelial_mesenchymal_transition, hypoxia, and TGF_beta_signaling. The pathway diagram of this GSEA shows that the C1 subtype is more related to tumors (Figure 3(f)).

### 3.3. A Comparison of Clinical Features between C1 and C2 Subtypes

In the TCGA dataset, the clinical characteristics in C1 and C2 molecular subtypes were compared to determine whether the clinical aspects differed in different subtypes. The results indicated that (1) the survival ratio of the two subtypes was significantly different, as the C1 group with a poor prognosis had a higher death rate; (2) there were no significant differences between the clinical features (stage, grade, and age of the C1 and C2 subtypes) (Figures 4(a)–4(d)).

### 3.4. Construction of a Prognostic Risk Model Based on Immune-Related lncRNA Pairs

#### 3.4.1. Identification of Differentially Expressed Immune lncRNA Pairs

We then used lncRNA to classify TCGA dataset. There was a noticeable difference in survival between the two subtypes. The prognosis of C1 was significantly lower than that of C2. Fisher's exact test was adopted to identify the differentially expressed lncRNAs between the subtypes, calculated the difference between the subtypes of each lncRNA pair, and then used the BH method to correct the corrected FDR for which a threshold of <0.05 was identified as a differential lncRNA pair. Thus, 180 differential lncRNA pairs were ultimately identified (Supplementary Table5).

#### 3.4.2. Random Grouping of the Training Set Samples

First, 373 samples from TCGA dataset were split into a training and testing set. Samples are grouped 100 times randomly by substitution. (training/testing set ratio = 7 : 3). The most suitable training set and testing set were selected in accordance with the following criteria: there was no statistical difference in clinicopathological factors (age distribution, gender, follow-up time, and patient mortality) between the two groups. The training set (261 samples) and testing set (112 samples) sample information of the ultimately obtained TCGA data are shown in Table 1. The results show that our grouping was reasonable, and that there was no significant variation between the two subgroups by the chi-square test (*p* > 0.05).

#### 3.4.3. Single- and Multifactor Risk Analyses of the Training Set

Using the training set data, for each differential lncRNA pair of C1 and C2 molecular subtypes (a total of 180) and the survival data, the R package survival coxph function was adopted to construct a univariate Cox proportional hazard regression model (*p* < 0.05 as a threshold), and 12 differential genes were analyzed. The univariate Cox analysis results were summarized in the Supplementary Table6.

Twelve different related lncRNA pairs were identified, but a large number of these lncRNA pairs were not conducive to clinical testing; therefore, we needed to further narrow the range of immune lncRNA pairs while maintaining a high accuracy rate. We used LASSO regression to compress these 12 lncRNA pairs further to reduce the number of lncRNA pairs in the risk model. First, we analyzed the change trajectory of each independent variable (Figure 5(a)). As the lambda gradually increased, the number of independent variable coefficients gradually tended to 0. We then used 5-fold cross-validation for model construction and analyzed the confidence interval under each lambda (Figure 5(b)), and when lambda = 0.0147, the model reached the optimal level. Thus, ten lncRNA pairs were used as the target lncRNA pairs in the next step.

The AIC Akaike information is used as a stepwise regression criterion, which refers to the statistical fit of the model and the number of parameters used to fit the model. The stepAIC method in the MASS package starts with the most complex model and deletes one variable to reduce the AIC. The smaller this value is for a model, the better the model, which means that the model uses fewer parameters to obtain a sufficient degree of fit. Using this algorithm, we ultimately reduced the 10 lncRNA pairs to 8 lncRNA pairs: lncRNA pairs AC027130.1_vs_AL391422.3, MRVI1_AS1_vs_AL391422.3, AC092198.1_vs_AC135012.2, AC016831.5_vs_AC104462.2, KIAA2012_AS1_vs_AC608.1_vs_AL391422.3, AC106037.2_vs_AL391422.3, and AL390208.1_vs_AL391422.3. It can be demonstrated from the prognostic KM curve that the eight pairs of lncRNA can remarkably separate the two groups of TCGA training set samples (Figure 5(c), *p* < 0.05). The final RiskScore formula was as follows: RiskScore = (−0.328∗AC027130.1_vs_AL391422.3) + (−1.457∗MRVI1_AS1_vs_AL391422.3) + (−0.488∗AC092198.1_vs_AC135012.2) + (−0.344∗AC016831.5_vs_AC104462.2) + (−0.364∗KIAA2012_AS1_vs_AC093843.1) + (0.749∗AC007608.1_vs_AL391422.3) + (−0.439∗AC106037.2_vs_AL391422.3) + (−0.995∗AL390208.1_vs_AL391422.3). There are 12 lncRNAs in these 8 lncRNA pairs. We extracted the expression profiles of 12 lncRNAs in these 8 lncRNA pairs from TCGA dataset and analyzed the expression distribution of these lncRNAs in C1 and C2 samples. It can be observed that MRVI1-AS1 is significantly overexpressed in C2, and AC016831.5, AC104462.2, and AC007608.1 are significantly overexpressed in C1 (Supplementary figure 1A). Combined with the overall survival data of patients, the relationship between these 12 lncRNAs and overall survival was evaluated by univariate survival analysis. The high expression of AC104462.2 and AC093843.1 was associated with poor prognosis (Supplementary figure 1B). In addition, we also analyzed the relationship between these lncRNAs and immune cell infiltration. It was observed that AC007608.1, AC104462.2, and AC106037.2 were significantly positively correlated with multiple immune cell infiltration (Supplementary figure 1C).

### 3.5. Construction and Validation of Risk Models

The risk score of each sample was analyzed in terms of the expression level of the sample and used the R software package time ROC to perform the ROC analysis of the prognostic classification of the RiskScore. The prognostic prediction classification efficiencies of one, three, and five years were calculated (Figure 6(a)). Finally, we analyzed the *z*-scores of the RiskScores, divided the samples with RiskScores greater than or less than zero after *z*-scorization into high- and low-risk groups, respectively, and drew a KM curve (Figure 6(b)). It can be indicated that they were very significantly different (*p* < 0.001), wherein 144 samples were classified as being in the high-risk group, and 117 samples were classified as being in the low-risk group.

In order to verify the robustness of the risk model, TCGA testing set and all TCGA_OV datasets (same model and coefficients as the training set) were applied to calculate the risk score of each sample per the expression level of the sample and drew the RiskScore distribution. The RiskScore of TCGA testing set was calculated, and we further used the “timeROC” package to perform the ROC analysis of the prognostic classification of the RiskScore. We analyzed the prognostic prediction classification efficiencies at 1, 3, and 5 years (Figure 6(c)). Finally, we calculated the *z*-scores of the RiskScores. After *z*-scorization, samples were divided into the high-risk group (RiskScores > 0) and low-risk group (RiskScores < 0), and the KM curve is drawn (Figure 6(d)). It can be suggested that they have incredibly significant differences (*p* < 0.05), of which 55 samples in the high-risk group and 57 samples in the low-risk group.

The RiskScores of all TCGA datasets were calculated using the same method as above. The model had a very high area under the AUC line (Figure 6(e)); the KM curve showed that they had a very noticeable difference (*p* < 0.0001), of which 199 samples in high-risk and 174 samples in low-risk (Figure 6(f)).

### 3.6. Correlation of RiskScores with Clinical Characteristics and Immune Scores

We compared the distribution of RiskScores among clinical feature groups and found that between the grade and age groups, there were no remarkable disparities between the RiskScore groups (Figures 7(b) and 7(d); *p* > 0.05), while there were notable disparities between stage and our classification groups (Figures 7(a) and 7(c); *p* < 0.05). In the middle to late stages, the RiskScores were higher (Figure 7(a)); in the classification grouping samples, the RiskScore of the C1 subtype with a poor prognosis was remarkably higher than that of the C2 subtype (Figure 7(c)). We used ESTIMATE, TIMER, ssGSEA, MCPcounter, and CIBERSORT to analyze the immune score of each sample and then calculated the correlation between these scores and the RiskScore. The results revealed that there was no apparent correlation (Supplementary Table7).

### 3.7. Identification and Functional Analysis of Related Genes by Model lncRNAs

We identified 8 model prognostic lncRNA pairs. We calculated the Spearman correlation coefficients between these lncRNA pairs and mRNAs and their significance. After filtering by the thresholds Corr > 0.3 and *p* < 0.05, we identified 351 genes (Supplementary Table8). Then, WebGestalt R (v0.4.2) was adopted to applicate KEGG pathway analysis and GO function enrichment analysis on the 351 genes. For the GO function annotation of the 351 genes, 186 items with significant differences in BP were annotated (FDR < 0.05, Figure 8(a)), 19 items with significant differences in MF were annotated (FDR < 0.05, Figure 8(c)), 27 were annotated with significant differences from CC to CC (FDR < 0.05), and the annotation results for the first 15 items were annotated (Figure 8(b)). For the KEGG pathway enrichment of the 351 genes, 11 significant entries were annotated (FDR < 0.05). The annotation results are shown in Figure 8(d) and included significant enrichment in proteoglycans in cancer, the PI3K-Akt signaling pathway, focal adhesion, ECM-receptor interaction, and other tumor-related pathways (Supplementary Table9).

### 3.8. Univariate and Multivariate Analysis of RiskScore

In order to determine the independence of the RiskScore model in medical application, the single- and multifactor Cox regression was used to calculate the relevant HR, 95% CI of the HR, and *p* value from the entire TCGA dataset. In TCGA dataset, we figured that RiskType was significantly related to survival in single-factor Cox regression analysis, and RiskType (HR = 1.9, 95%CI = 1.44–2.5, and *p* < 1*e* − 5) was still significantly related to survival in multivariate Cox regression analysis. These results clarified that the RiskScore model has excellent prediction in terms of clinical application value (Figures 9(a) and 9(b)).

### 3.9. Construction of a Nomogram and DCA Curve with RiskScore and Clinical Characteristics

The nomogram can be a more intuitive and effective way to display the outcomes of the risk model and is more convenient to apply in predicting outcomes. The nomogram uses straight lines to suggest the degree of influence of distinct variables and the influence of different values on the outcome. We built the nomogram model together with the clinical features age and RiskScore, and we used all TCGA datasets to create the nomogram (Figure 10(a)). The RiskScore feature had the greatest impact on the survival rate prediction from the model outcomes, hinting that the lncRNA pair-based risk model could better predict the prognosis. In addition, we corrected the nomogram data for 1, 3, and 5 years to visualize the performance of the nomogram (Figure 10(b)), which proved that the method had a good performance. We then drew the DCA diagrams for age, RiskScore, and nomogram. The results showed that our RiskScore had a good effect, and the nomogram had a better outcome (Figure 10(c)).

### 3.10. Correlation Analysis of the Risk Model, Immune Checkpoint Genes, and Chemotherapy Drugs

We compared the expression differences of CTLA4, PDCD1, CD274, CD276, TNFSF4, and TNFRSF18 in the high- and low-risk groups and indicated remarkable differences between the high- and low-expression groups (Figure 11(a)). In TCGA project of the OV dataset, we also tried to determine the correlation between RiskScore and the efficacy of general chemotherapy for OV using pRRophetic to predict the drug sensitivity of each sample. The results showed that paclitaxel and dasatinib in the high-risk group had lower IC50 values (*p* < 0.05), while saracatinib and parthenolide had higher IC50 values. These results indicate that the model can be used as a potential predictor of chemical sensitivity (Figure 11(b)); to compare the superiority of our RiskScore with clinical characteristics, we used all TCGA datasets to draw the ROC curve, and the results showed that our RiskScore had the largest AUC value, proving that our RiskScore is superior to other clinical features (Figure 11(c)).

## 4. Discussion

Increasing evidence indicates that the immune system displays an essential role in tumor development [28]. Immunotherapy is a treatment method that enhances the autoimmune ability of patients to kill or eliminate OV cells [29]. It includes various forms, such as tumor vaccines and immune cell therapy [30, 31]. As an essential means of tumor treatment, tumor immunotherapy can achieve the purpose of therapy by regulating tumor immunity through noncoding RNA [32]. Previous prognostic risk models are needed to properly standardize gene expression profiles in view of the inherent biological heterogeneity of tumors and the technical deviations brought about by different sequencing platforms [33]. In order to accomplish the robustness of the forecast, we evaluated a new method for data analysis without considering the technical deviations of different platforms. The novel established prediction method does not require data preprocessing (scaling and normalization) but is mediated by relative ranking and pairwise comparison of gene expression values.

As mentioned in the literature review, Nie et al. indicated 29 IRGPs as crucial gene pairs and established a cervical cancer model, which can serve as a prognostic biomarker and potential novel target [34]. Wu et al. constructed a 19-IRGP signature (a total of 36 unique genes) that was significantly relevant to survival in CRC, presenting new strategies for identifying CRC patients with a high risk of mortality [35]. Zhang et al. constructed a robust IRGP signature with prognostic value for serous OV, presenting novel insights into postoperative treatment strategies [36]. The method of gene relative rank can effectively avoid the result deviation caused by different data processing and standardization between different datasets. This method has obtained reliable gene pair-based outcomes in studies. In comparison, there have not been systematic reports of immune-related gene pairs based on lncRNAs.

Noncoding RNA serves a vital role in the tumorigenesis and development of tumors: it can promote chromatin modification; mediate gene silencing, act as a protein guide molecule and scaffold to promote the formation of cell substructures, control protein synthesis, and RNA maturation, and transportation [37], and competitively bind to miRNA, reducing the regulatory effects of a miRNA on its target RNA [38]. Therefore, we constructed an immune-related lncRNA gene pair (IRLnc_GP) prognostic model by screening for IRGs significantly related to prognosis and verified the model. The 373 OV samples were divided into two IRLnc GP subtypes (C1 and C2). IRLnc_GP typed 373 OV samples of TCGA (C1 and C2 subtypes). The subtypes showed significant differences in prognosis. By calculating the Spearman correlation coefficients between 8 IRLnc_GPs and mRNAs, which were significant for sex, we obtained 351 genes. Further enrichment analysis found that hypoxia, TGF-*β* signaling pathway, proteoglycans in cancer, focal adhesion, PI3K-Akt signaling pathway, Wnt_beta_catenin signaling pathway, and other tumor-related pathways were statistically significant enriched. Previous studies [24] have found that the activation of the JAK/STAT pathway plays an essential role in the immune escape, especially the STAT3 molecule, which not only can increase the expression of inhibitory cytokines such as VEGF, IL-6, IL-10, and TGF-*β* but can also be activated by these cytokines to enhance their own activity. STAT3 inhibits the maturation of DCs, promotes the accumulation of Tregs, induces an immunosuppressive microenvironment, inhibits the killing effect mediated by NK cells and neutrophils, and jointly promotes tumor cell immune escape [39, 40]. The TGF-*β* signaling pathway can inhibit glycolysis in NK cells, leading to low activity of NK cells in the tumor microenvironment, thereby mediating immune escape. In addition, MAPK, NF-*κ*B, PI3K/AKT, and other pathways are activated in a variety of tumors, which together promote the generation and progression of the immunosuppressive inflammatory microenvironment [41]. The C1 subtype with a poor prognosis is more related to the pathways of tumor occurrence and development, which may explain why the C1 subtype has a poor prognosis. In the future, the prognosis of patients with the C1 subtype may be able to be improved by further in-depth research. In addition, single-factor, multifactor, and nomogram analyses show that the risk model based on IRLnc_GP has good predictive performance in clinical applications. In independent datasets, the distribution of subtypes in functional modules is different, and the results are highly repeatable.

Immune checkpoint inhibitors also play a critical role in tumor treatment. This immunotherapy method has been clinically applied in various tumors, such as melanoma [42], non-small-cell lung cancer [43], and Hodgkin's lymphoma [44]. There are research reports that targeting immune checkpoints such as programmed cell death ligand 1 (PD-L1) and programmed cell death receptor 1 (programmed cell death protein 1, PD-1) has a significant correlation between immunotherapy and the prognosis of OV [45]. Through the analysis of the correlation between the risk model and immune checkpoint genes and chemotherapy drugs, we compared the expression differences of common immune checkpoints (CTLA4, PDCD1, CD274, CD276, TNFSF4, and TNFRSF18) in the high- and low-risk groups. From the significant differences, the association analysis between RiskScore and the efficacy of general chemotherapy for OV showed that paclitaxel, saracatinib, dasatinib, and parthenolide in the high-risk group have low IC50 values, indicating that this model can be used as a potential chemosensitivity predictive index.

The study results indicated that the combination of PD-1 inhibitors, the cytokine IL-2, and immune cell therapy could successfully cure patients with advanced OV [46]. The abovementioned studies point out the direction for the comprehensive treatment of tumors. To compare the superiority of our RiskScore with clinical features, we used the entire TCGA dataset to draw the ROC curve. The results showed that our RiskScore had the largest AUC value, proving that our RiskScore is superior to other clinical features (Figure 11(c)).

## 5. Conclusion

We have systematically studied the value of IRGP markers in the prognosis of OV patients to provide a risk assessment for OV treatment. The biological functions of these immune marker genes provide a basis for further understanding the roles of the prognostic markers in the development of OV.

## Figures and Tables

**Figure 1:** Prognostic schemes related to the characteristics of immune gene-related lncRNA pairs in OV.

**Figure 2:** (a) Map showing NMF Clustering Consensus. (b) Cophenetic, RSS, and dispersion distributions with rank = 2‐10. (c) OS time prognostic survival curve for OV molecular subtypes. (d) Curve of prognosis for OV molecular subtypes according to PFS time.

**Figure 3:** (a) Comparison of ssGSEA immune scores between the C1 and C2 groups. (b) Assessment of MCPcounter immune scores between the C1 and C2 groups. (c) Comparison of ESTIMATE immune scores between the C1 and C2 groups. (d) Comparison of TIMER immune scores between the C1 and C2 groups. (e) Comparison of CIBERSORT immune scores between the C1 and C2 groups. (f) Related pathways between molecular subtypes.

**Figure 4:** (a–d) Comparison of the distribution of different clinical characteristics (event, grade, stage, and age) between the two molecular subtypes in TCGA dataset.

**Figure 5:** (a) The changing trajectory for each independent variable. The logarithm of the independent variable lambda is shown on the horizontal axis, and the coefficient of the independent variable is represented by the vertical axis of the graph. (b) The confidence interval for each lambda. (c) The 8 lncRNAs vs. the KM curve (on TCGA training set).

**Figure 6:** (a) ROC curve and AUC of RiskScore classification. (b) Survival curves for RiskScores calculated using KM in the training set. (c) ROC curve and AUC of RiskScore classification. (d) KM survival curve distribution of RiskScore in TCGA test set. (e) ROC curve and AUC of RiskScore classification. (f) KM survival curve distribution of RiskScore in all TCGA datasets from TCGA.

**Figure 7:** (a) Comparison of RiskScores between samples in the stage group. (b) Comparison of RiskScores between samples in the grade group. (c) Comparison of RiskScores between samples in the cluster group. (d) Comparison of RiskScores between samples in the age group.

**Figure 8:** (a) BP annotation map of lncRNA to genes. (b) CC annotation map of lncRNA to genes. (c) MF annotation map of lncRNA to genes. (d) KEGG annotation map of lncRNA to genes.

**Figure 9:** (a) Clinical characteristics and RiskScore single-factor analysis results. (b) Clinical characteristics and RiskScore multifactor analysis results.

**Figure 10:** (a) Clinical features and risk-adjusted nomogram developed using RiskScore. (b, c) Nomogram of the survival rate correction chart.

**Figure 11:** (a) Expression of immune checkpoint genes in the low- and high-risk groups. (b) Comparison of drug sensitivity between the low- and high-risk groups. (c) Clinical characteristics and the RiskScore ROC curve.

**Table 1:** TCGA training and validation set sample information.

Clinical features	TCGA train	TCGA test	*p*
OS			
0	102	41	0.7383
1	159	71	
Stage			
I	0	1	0.3699
II	17	4	
III	205	86	
IV	37	20	
X	2	1	
Grade			
G1	0	1	0.3094
G2	29	13	
G3	226	93	
G4	1	0	
GX	5	5	
Age			
≤60	143	61	1
>60	118	51	

## Data Availability

Upon a reasonable request, the datasets used and/or analyzed in this investigation may be obtained from the corresponding author.

## Supplementary Materials

Supplementary 1 Supplementary Figure 1: expression relationship of 12 lncRNAs in 8 lncRNA pairs. (A) The expression and distribution of 12 lncRNAs in C1 and C2 subtypes were different. (B) Univariate survival analysis forestplot of 12 lncRNAs. (C) Correlation between the expression of 12 lncRNAs and immune cell infiltration.

Supplementary 2 Supplementary Table 1: a total of 373 preprocessed TCGA-OV sample information.

Supplementary 3 Supplementary Table 2: 260 lncRNAs and 246 IRGs.

Supplementary 4 Supplementary Table 3: TCGA lncRNA pair data were analyzed, and 426 lncRNA pairs were obtained.

Supplementary 5 Supplementary Table 4: the 51 enriched pathways were selected.

Supplementary 6 Supplementary Table 5: 180 differential lncRNA pairs were identified.

Supplementary 7 Supplementary Table 6: the univariate Cox results of the training set were summarized.

Supplementary 8 Supplementary Table 7: the immune score of each sample and the correlation between scores and the RiskScore.

Supplementary 9 Supplementary Table 8: 351 genes were identified by the Spearman correlation coefficients.

Supplementary 10 Supplementary Table 9: enrichment analysis and tumor-related pathways.
